RETRACTED

# Beliefs and Practice Evaluation Based on Artificial Intelligence Models under the IP Environment

**DOI:** 10.1155/2022/1415142

**Published:** 2022-09-27

**Authors:** Yang Zhou

**Affiliations:** School of Marxism, Zhengzhou College of Finance and Economics, Zhengzhou 450000, China

## Abstract

The digitization of thought theory is not yet sufficient to meet the needs of the students. It is very necessary to strengthen the construction of ideological and political (IP) courses, strengthen the education of mainstream ideology, and occupy the initiative of discourse. There are effective ways and means to study the deep integration of information technologies into the new age of philosophy and philosophy education of students, which can greatly improve the quality of teaching and the effectiveness of humanities courses. The intuitive development of intellectual and political education through artificial intelligence is both a real prerequisite for modern development and technological innovation and for new ideas confronting the specific problems of thought-politics education, and it is a necessary prerequisite to ensure the quality and efficiency to improve the teaching of thought politics. AI in ways that embed technology provides a powerful impetus for contradictory movements in thought-politics discourse that lead the effective coordination of its internal elements to high-quality developments. In a practical way, we should take full advantage of the technical advantages of artificial intelligence, through intelligent mehrfachanalyse corresponding algorithms, artificial intelligenzbilder, and artificial roboterbilder photos and profiles that are used to write and accurately provide more precise, leading, stacking, and accurate estimates to maximize and to improve the accuracy of thought and policy education. Philosophy and political theory are the keys to guiding people to accomplish basic human tasks. With the passage of time and with continuous innovation, ideology and philosophical principles are both prerequisites for the self-development of the emotions of the age and necessary for improving the outcomes and effectiveness of scientific education. Advances in the field of artificial intelligence have fundamentally changed human life and have also impacted traditional school and university education systems. This brings new opportunities and challenges to students. This includes the use of smart technology to improve the learning process. Ideological teachers and policymakers must keep up with the all-round trend of the times, make full use of the benefits brought by intelligent new technologies and platforms, effectively improve the effect of ideological education, and further increase the attractiveness, attraction, persuasion, and contagion of ideological education.

RETRACTED

## 1. Introduction

Artificial intelligence is concerned with the development of systems, or intelligent machines, that simulate human activities, thereby expanding the science of human intelligence. In 2016, the research in Alphago and Lee's Dragon robot will rise to a new peak. A new year of artificial intelligence will result. In recent years, artificial intelligence development has been integrated into China's national strategy [1]. In 2017, “artificial intelligence” was included in the government report for the first time, which gave: the new AI development planning, requires the intelligence education, “use intelligent technology to accelerate the culture-specific teaching and learning methods, build intelligence and interact learning new, the intelligence campus, promote AI, and, management, resources structure. As shown in Figure 1, AI is a broad concept, including deep learning. The continuing breakthroughs in critical technologies such as autonomous learning adaptation, deep learning, computer vision, natural language understanding, and virtual reality will drive new trends in instruction, method, methodology, and the role of the teacher [2]. In the book, ideological theorists deepen the innovation in the field of philosophy textbook reform in the new era. it becomes clear that it is necessary to “improve the ability and competence of the idea-oriented teachers and the application of modern information technologies, such as of artificial intelligence in teaching ideas on politics”. It vigorously promotes the reform of teaching methods of IP courses, improves the informatization ability and quality of IP curriculum teachers, promotes the application of modern information technology such as artificial intelligence in IP curriculum teaching, and builds a number of national-level virtual simulation experience teaching centers for IP courses. This provides a guide to artificial intelligence-based thought-politics courses [3]. Artificial intelligence improves the absorbency of teaching in colleges and improves the effectiveness and appeal of teaching, but artificial intelligence is still in its infancy [4]. There are many difficulties in integrating politics and schools of thought into schools. Thought-politics teachers must face challenges objectively, respond boldly, and find reasonable ways and means to effectively improve the effectiveness of artificial intelligence thought education reform.

It has become an important direction for the development of education to promote the integration of education and artificial intelligence and to promote the high fit between education supply and students' needs [5]. For the teaching of political thought courses, promoting the deep integration of artificial intelligence and teaching is not only an inevitable trend to comply with the development of science and technology [6] but also a self-need to promote teaching accuracy, enhance teaching efficiency, and improve teaching pertinence. The technology embedding of artificial intelligence provides a strong driving force for the contradictory movement of IP teaching, drives the precise docking and efficient coordination of its internal elements, promotes the high-quality development of IP teaching in the direction of precision, and thus provides a new picture for solving the practical problems of IP teaching. However, most of the political thought teachers in China have a short teaching experience (Figure 2), and their acceptance of AI technology varies. The basic assumption of intelligent political thought education [7] is to embed and integrate advanced and appropriate new generation information technology into the political thought theory teaching and make it as an endogenous variable to drive the political thought theory teaching idea renewal, paradigm transformation, and system reform, so as to ensure the orderly and efficient development of the political thought theory teaching and strive to cultivate the ideological level, political awareness, and moral quality. A comprehensively developed socialist builder and successor meets the needs of the times in terms of cultural literacy [8].

RETRACTED

Political thought teachers should further consolidate and give play to their unique advantages and charm in the artificial intelligence environment [9], educational content, and educational methods, and educators play a leading role in the process of political thought education.  Figure 3 describes the distribution of cultural literacy of political thought teachers in China. It can be seen from the figure that most political thought teachers have a bachelor's degree or above. The political thought education system is a rigorous and complete system, and the lack of any factor will lead to the overall operation of the whole is not smooth, not to mention the important role of educators who play a leading role in this process is self-evident [10]. This is not only caused by the limitation of technology itself but also the embodiment of the unique “educating” advantage of political thought course teaching. Artificial intelligence will replace a lot of mechanical repetitive work of political thought teachers, such as question answering guidance [11], homework correction, and test paper analysis and help them save a lot of time and devote more energy to enlightening and personalized teaching. However, no matter how developed the artificial intelligence is, it is always based on the established knowledge and does not have the ability to actively create new knowledge. It is unable to cultivate contemporary college students to form correct values, moral character, and profound cultural heritage. Political thought teachers should actively overcome this defect of artificial intelligence and give full play to their dominant advantages [12]. They should use the development of technology to solve some problems in “teaching” and help students acquire political thought-related knowledge faster and better [13]. On the other hand, they should bear the historical responsibility of “educating people.” They should strive to become students' spiritual tutors through words and deeds, cultivate students' wisdom, inspire students' minds, and help students establish a scientific world outlook, outlook on life and values.

RETRACTED

## 2. Limitations of Traditional Political Thought Teachers' Teaching Beliefs and Teaching Practices

With the integration of natural science and social science and the rise of “new liberal arts,” the future society needs compound talents with data literacy, cultural literacy, learning ability, and innovation ability [14]. However, due to the professional complexity of artificial intelligence technology, it is difficult for IP teachers to reasonably use intelligent tools in a short time, and it is easy to be interfered with the teaching ideas by the artificial intelligence technology, which makes it difficult to implement the artificial intelligence technology in the teaching process. Teachers, as guides of education and teaching, should cross the digital divide and actively develop their own information literacy. Artificial intelligence can generate a comprehensive and three-dimensional visual knowledge map according to the ideological dynamics, learning mode, and interpersonal communication status of different educated individuals. If political thought teachers do not pay attention to the transformation of thinking mode, when using the visual knowledge map, and still adhere to the traditional teaching thinking, they may be disturbed by redundant digital images and cannot effectively play the role of artificial intelligence [15]. The level is relatively shallow. Classroom teaching and student evaluation feedback and other links have not been innovated due to the application of artificial intelligence technology. Therefore, it is urgent for political thought teachers to cooperate with AI technology and fully improve teachers' ability to use technical tools, promote the collaborative education process of artificial intelligence and political thought courses, and then guide students to achieve the mastery of learning, thinking, and using and the unity of knowledge, belief, and practice [16]. Political thought course is a key process to solve the fundamental problem of who, for whom, and how to cultivate people. It is a teaching activity of guiding values, imparting knowledge and cultivating ability around the two interrelated subjects. The understanding and application of artificial intelligence technology is an innovative thinking about political thought courses. However, due to the generalization effect of technical rationality and data collection presented by intelligent algorithms, the attention to human inner empathy is ignored, and the subject richness of political thought teachers and students is eliminated. On the one hand, the personification of human-computer interaction leads to the desolation of the subjectivity of political thought teachers [17]. The integration of artificial intelligence into political thought courses is a process in which artificial intelligence technology is used as an auxiliary tool to enlarge the effectiveness of education according to the will and instructions of teachers in the field of modern information technology [18]. However, artificial intelligence has the attribute of human brain, which is not a physical machine in the general sense. It is very easy to appear the exclusivity of technology and then dispel the value rationality of teachers. With the development of human-computer interactive learning, artificial intelligence is more likely to win the attention of educators when it improves the classroom effect, reversing the order of education oriented and tool assisted, thus gradually weakening the guiding role of teachers as the main body of political thought courses. On the other hand, it dispels students' subjective initiative. Artificial intelligence can provide students with the technical support of “automatic supply of learning question answers” based on early data analysis, and the acquired knowledge also shows the characteristics of one-sided and fragmented [19]. And most of the information pushed is to coerce vulgar content information in a playful way of expression, imperceptibly reshaping students' way of thinking and cognitive schema, resulting in students' narrow vision, information persistence [20], falling into the dilemma of information cocoon, and difficult to carry out knowledge innovation and academic exploration, and the brain and thinking are increasingly materialized. We must ensure the subjectivity of witnesses and the instrumental status of intelligent technology, build a personalized teaching platform, implement differentiated guidance, and enrich classroom teaching models [21].

RETRACTED

Practical teaching is a teaching activity that enables students' ideas to interact deeply with the external environment through problem discussion, in-depth experience, critical reflection, and other practical forms and enhances their understanding of the objective world and theoretical knowledge in this process [22]. In the teaching of IP theory, the core function of practical teaching is to further strengthen the students' belief in Marxism, consolidate the correct world outlook, outlook on life and values, and enable them to master and learn to use Marxist theoretical weapons and methods. However, in practice, the proportion of practical teaching is not high (Figure 4). But on the whole, practical teaching is not only highly valued in practical teaching activities [23] but also often a difficulty in the teaching system. There are still some prominent problems in the practical teaching of political thought courses under the traditional mode, which restrict the fundamental and sustainable improvement of teaching effect.

Flexible form was originally an important feature that distinguishes practical teaching from classroom teaching, but in actual teaching activities, some schools and courses did not deeply explore the laws of practical teaching activities, and the selection of practical teaching methods was not detailed and reasonable, resulting in simple response and uniformity in the organization of practical teaching. The disadvantage of these methods is that they are difficult to combine with the real social situation [24]. At most, participants can only understand and reflect on social phenomena or theoretical knowledge in their subjective imagination space. Off-campus practical teaching such as visiting and learning and social investigation is relatively closer to the real situation, and it is easy to stimulate students' interest, but it is often subject to defects such as difficult organization and implementation, difficult safety assurance [25], and difficult assessment and evaluation, so the actual teaching is less carried out or the effect is poor.

Students are the cognitive subjects of objective laws, scientific truth, and values. There are difficulties in organizing diversified practical teaching activities and other factors, the embodiment of students' dominant position in practical teaching is not obvious, and most of them passively complete the established tasks arranged by teachers, such as watching specific video materials and publishing their experiences, so there is little space for students to actually explore [26], and some activities have become mere task-based walk through behavior.

RETRACTED

When some political thought courses are designed for practical teaching, they either do not understand what the students want to practice or understand the object of practice, but there is no appropriate way to implement it, resulting in a relatively general teaching design as a whole, and there is a lack of clear logical connection and goal orientation between methods and ability training. That is to say, before some practical teaching activities are carried out, teachers are not quite sure what practical abilities students can cultivate through this activity, and students do not know what abilities they should focus on in the activities, which is also part of the reason for the single teaching mode and other problems pointed out above. On the whole, there are some limitations in the practice teaching of IP theory under the traditional mode. In particular, it is difficult to form an organic unity between teaching methods and teaching objectives, which makes the enthusiasm and initiative of students participating in practice teaching not fully developed, and the effectiveness of teaching is also affected. The final result is that the complete closed loop from classroom knowledge teaching to practical ability training is not fully formed. To further improve the quality of political thought teaching, we should vigorously strengthen the exploration of practical teaching mode and seek the way of reform and innovation.

## 3. Research Methods and Models

The subjective Bayesian method is used to simulate the teaching beliefs and teaching practices of political thought teachers. A basic tool in Bayesian statistics is called “Bayesian rule.” Although this is a mathematical equation, its principle can be understood without numbers. If you see that a man always does the right thing, maybe he is a good man. That is, if the nature of a thing is not precisely known, the probability for a trait can be determined by the number of events related to that particular character of the thing. The more events that support a profile, the greater the likelihood that it will emerge.

Beatle's rule is also called Beth's theorem. This is Baeli's rule, a common way of applying probability statistics to correct the observational phenomenon of probability [27]. Some investors are not perfectly rational in their decision-making and judgement, leading to behavioral biases which in turn can affect price changes in the capital markets. However, in the absence of strong alternative tools, economists have long been forced to incorporate Baeli's law into their analyses.

In the subjective Bayesian method, knowledge is expressed by production rules, and the specific form is

(1) $$\begin{array}{c} \text{LS}=\frac{P\left(\left.E\right|H\right)}{P\left(\left.E\right|\neg H\right)}. \end{array}$$

(2) $$\begin{array}{c} \text{LN}=\frac{P\left(\neg \left.E\right|H\right)}{P\left(\neg \left.E\right|\neg H\right)}=\frac{1-P\left(\left.E\right|H\right)}{1-P\left(\left.E\right|\neg H\right)}. \end{array}$$

LS is called the sufficiency measure, which is used to indicate the support degree of *E* to *H*. LN is called the necessity measure, which is used to indicate the degree of *E*'s support for *H*. The values of LS and LN are given by domain experts, which are equivalent to the static strength of knowledge.

RETRACTED

*P*(*H*) is the prior probability of conclusion *H*, which is given by experts based on experience:

(3) $$\begin{array}{c} P\left(\left.H\right|E\right)=\frac{P\left(\left.E\right|H\right)\times P\left(H\right)}{P\left(E\right)}, \end{array}$$

(4) $$\begin{array}{c} P\left(\neg \left.H\right|E\right)=\frac{P\left(\left.E\right|\neg H\right)\times P\left(\neg H\right)}{P\left(E\right)}, \end{array}$$

(5) $$\begin{array}{c} \frac{P\left(\left.H\right|E\right)}{P\left(\neg \left.H\right|E\right)}=\frac{P\left(\left.E\right|H\right)}{P\left(\left.E\right|\neg H\right)}\times \frac{P\left(H\right)}{P\left(\neg H\right)}. \end{array}$$

The method of determining the posterior probability based on the known probability varies with the existence, nonexistence, or uncertainty of the evidence:

(6) $$\begin{array}{c} O\left(X\right)=\frac{P\left(X\right)}{1-P\left(X\right)}, \end{array}$$

(7) $$\begin{array}{c} O\left(X\right)=\frac{P\left(X\right)}{P\left(\neg X\right)}. \end{array}$$

The above formula is called the probability likelihood form of Bayes formula. LS is called sufficient likelihood. If LS > +∞, the evidence *E* is logically sufficient to deduce that *H* is true. Similarly, it can be obtained:

(8) $$\begin{array}{c} O\left(\left.H\right|E\right)=\frac{P\left(\left.E\right|H\right)}{P\left(\left.E\right|\neg H\right)}\times O\left(H\right). \end{array}$$

When the combined evidence is the combination of multiple single evidence, the probability is as follows:

(9) $$\begin{array}{c} O\left(\left.H\right|E\right)=\text{LS}\times O\left(H\right), \end{array}$$

(10) $$\begin{array}{c} \frac{P\left(\left.H\right|\neg E\right)}{P\left(\neg \left.H\right|\neg E\right)}=\frac{P\left(\neg \left.E\right|H\right)}{P\left(\neg \left.E\right|\neg H\right)}\times \frac{P\left(H\right)}{P\left(\neg H\right)}. \end{array}$$

When the combined evidence is the extraction of multiple single evidence,

(11) $$\begin{array}{c} O\left(\left.H\right|\neg E\right)=LN\times O\left(H\right). \end{array}$$

Finally, the relationship between probability and probability is as follows:

(12) $$\begin{array}{c} O\left(E\right)=\frac{P\left(E\right)}{1-P\left(E\right)}=\left\{\begin{array}{c} 0,\\ \infty ,\\ \left(0,\infty \right). \end{array}\right. \end{array}$$

Bayionists assign probabilities based on unknown propositions. One result is that bayionists have more opportunities to use Bayesian law. The operation process of subjective Bayesian method used in political thought teaching is shown in Figure 5.

RETRACTED

Heisani pointed out that all games with incomplete information under the old definition can be remodeled into a complete but imperfect information game without changing its essence, which only needs to add an initial action selected by nature in different rule sets. In the old definition, game theorists often pointed out that games with incomplete information are not analyzable, and Heisani's creativity has changed all this. The old definition is described as follows: in a complete information game, all participants know the rules of the game; otherwise, the game is an incomplete information game. Although Heisani did not point out that the old definition is problematic, in fact, people's views have changed, thinking that in the original definition, the game after conversion is incomplete information game. In the game, some participants may not be very clear about the payment of the game, but they still have a certain understanding of the payment. Generally, subjective probability distribution is used to represent information. That is, based on probability pairs, various game payments can be grouped to form a specific payment set. For example, when choosing strategies between a and B, it can be considered that when a chooses a certain strategy, B chooses several strategies, and these strategies of B are grouped according to the probability of occurrence. Usually, building a game tree can better express all this. The key point of the Heisani doctrine is to assume that all participants have a common understanding, and the probability of strategy adoption is a common knowledge. The implication is that participants' guesses about themselves are at least a little public.

When dividing the information structure of a game, we do not try to decide what participants can infer from the actions of other participants. Prior probability exists as a part of the game rules. Therefore, a participant must hold prior beliefs about other types of participants. At the same time, after observing their actions, it is necessary to assume that they follow balanced behavior, and then update their beliefs. Theoretically, it looks perfect, but in practice, it cannot be used directly. Therefore, we will make some assumptions in many classification methods to approximate the requirements of Bayesian theorem.

RETRACTED

## 4. Results and Discussion

### 4.1. Artificial Intelligence Drives the Basic Principles of Teaching Belief and Practice of Political Thought Teachers

The innovation of the teaching mode driven by artificial intelligence can improve the unity of teachers' ideological form and science.  Figure 6 shows the familiarity of political thought teachers with the basic principles of teaching practice.

The teaching process of political thought courses driven by artificial intelligence not only has the commonness of general courses but also has its own unique attributes, that is, to teach students scientific knowledge, with strict scientificity and knowledge. At the same time, it has a distinct value orientation, reflecting a strong political and ideological nature [28]. The unity of ideology and scientificity is the fundamental expression of its inherent unity. The reason why we should adhere to the unity of ideology and scientificity is that things are always moving and developing and cannot remain unchanged. Closed and backward ideas will only lead to the transformation of ideas from science to nonscience. Discipline and integrity are unified [29]. The unity of discipline and integrity is deeply contained in the integration of artificial intelligence and political thought teaching. On the one hand, we should refine the new direction of discipline construction. The teaching mode of political thought courses enabled by artificial intelligence will evolve into a complex dynamic system, which also marks the gradual transformation of the curriculum system of political thought courses driven by artificial intelligence from a single dimension to interdisciplinary and multidisciplinary. With the further integration of artificial intelligence technology and IP teaching, the analytical logic, data collection methods, learning scene applications, and teaching methods of the IP teaching mode will be strengthened correspondingly, and the coordination and integration of various disciplines will be further improved. On the other hand, the embedding of artificial intelligence can enable political thought education to grasp the integrity between different courses and within the same course. At the same time, it can grasp the actual differences and characteristics of teachers and students from a macroperspective, carry out targeted classification and aggregation, and measure the effects fed back by different types and educational subjects and objects, so as to obtain a holistic conclusion [30]. At the same time, we can also consider all links of teaching model innovation as a whole, so as to guide the collaborative innovation and application of political thought teaching among multiple disciplines. The calculation and measurement tools based on artificial intelligence technology can effectively mine and deeply analyze all kinds of information generated in the practice of political thought education. Through the extraction and adaptation of words, symbols, audio, video, etc. generated in the information, we can fully understand the needs of teaching subjects and objects, so as to form data integration and find appropriate teaching programs. This will greatly improve the pertinence of the political thought education model. At the same time, artificial intelligence technology is also reshaping the process of political thought education mode [31]. The cloud platform based on data integration can easily capture teaching information and evaluation data and clearly understand students' interest orientation and learning habits (as shown in Figure 7), and accurate push and personalized teaching services are beginning to be recognized by political thought teaching classes.

RETRACTED

In addition, AI technology also has a profound impact on the governance process of political thought education in the traditional sense. Through the crawling and homing of information, we can carry out targeted data analysis on the audience of political thought education, achieve accurate portraits, and provide more accurate teaching services for teachers and students with different cognitive abilities and acceptance levels, which can greatly expand information channels and improve information energy efficiency. It also fundamentally ensures the effectiveness of political thought teaching. Initiative and regularity are unified. The innovation of the teaching mode of political thought courses should not only rely on the technical advantages of artificial intelligence [32] and give full play to the subjective initiative of the subjects of political thought courses but also give full play to the advantages of artificial intelligence in intelligence, interaction, accuracy, and rapidity through data mining of existing cloud services, Internet of Things, intelligent systems, and other applications and organically combine political thought education with artificial intelligence technology, which is the main position for the publicity of socialist core values. IP courses have political attributes and follow the laws of political operation. It has scientific attribute and follows the law of academic research. It has educational attributes and follows the laws of education and teaching and forms a symbiotic development path with complementary functions, interdependence, and mutual support.

RETRACTED

### 4.2. The Implementation Strategy of Artificial Intelligence Driving Teaching Belief and Teaching Practice of Political Thought Course Teachers

The era of intelligence is the time and trend that political thought courses must firmly grasp. Intelligent technology and its application provide a new field for the transformation of political thought education from theory to practice. Only by actively using all kinds of intelligent platforms to broaden the ways, enrich the means, and enrich the connotation of practical teaching activities of political thought courses can we better promote the innovation and development of political thought teaching.

To realize the interactive teaching in the algorithm recommendation field, we need to improve the quality of interactive content from two aspects. On the one hand, teachers should be alert to algorithm power, improve their theoretical literacy, scientific research level, and algorithm literacy, and enhance the political height, theoretical depth, and discourse temperature in the selection of political thought course content [33]. Pay attention to the combination of social hot spots, theoretical knowledge, and students' reality, guide students to analyze current hot spots through interactive teaching, and improve the theoretical depth and problem-solving ability. On the other hand, teachers should improve their screening ability and improve the consistency between the algorithm recommended content and the interactive content of political thought courses. The teaching content system of the IP course is complete and the content is consistent. The content recommended by the algorithm has the characteristics of fragmentation, timeliness, personalization, and pan entertainment, but the quality of the content is mixed. This requires political thought teachers to have strong theoretical and algorithmic literacy, optimize interactive content, master students' real-time situation through big data analysis, evaluate the content of interest to students, and guide students to discuss current social hot issues with critical thinking to achieve interaction. In line with students' interests and close to the reality of students' life, it is more important to give full play to the role of political thought courses in cultivating morality and talents and guiding students to grow and become talents. The development of information technology and intelligent algorithm technology requires political thought teachers to have not only theoretical foundation but also information literacy when controlling interactive teaching and designing interactive teaching mode. Interaction is not a simple question and answer, but through “question chain,” “case base,” “interactive field,” and other forms of change and innovation [34]. In view of the impact of the algorithm, teachers can throw out the “algorithm dispute” problem, guide students to view the push content received in their mobile apps, and think about and discuss the advantages and disadvantages of the algorithm, so as to view the algorithm rationally. The “problem chain” should highlight the problem logic and guide students to think and discuss through open-ended questions and linked forms, so as to introduce special theoretical knowledge and realize the unity of value and knowledge. The “case base” teaching mode is the iteration of the case method in the era of algorithm recommendation, that is, to master the cases and topics of interest to students through the algorithm database and then select the classic and latest cases to form a case base suitable for each class and group for interactive teaching. “Interactive field” is based on algorithm recommendation, which not only requires offline classroom interaction but also extends the field of teaching interaction to online and extracurricular. Online interaction can combine various social media platforms, teaching interaction platforms, and other platform resources. Extracurricular interaction is based on the concept of “great political thought interaction,” which extends political thought interaction to social life, so as to arouse students' thinking, guide students from paying attention to pan entertainment content to paying attention to social conditions, and cultivate feelings of home and country. The development of intelligent algorithm provides technical support for interactive classroom interaction platform and can choose personalized learning platform according to the specific characteristics of students. Build a multidimensional three-dimensional teaching platform of virtual simulation and human-computer interaction. At the same time, with the help of AR, VR, and other auxiliary software and hardware facilities, students can personally participate in the classroom and scene through immersive scene experience, so as to strengthen emotion and value recognition. Based on the characteristics of the era of intelligent media, audio-visual resources are developed, respectively, in combination with the data recommended by the algorithm, so as to achieve full coverage and accurate dissemination of teaching content. At the same time, combined with the back-end data of the political thought course intelligent platform and the data of the learning terminal, we can realize the whole process recording and analysis of students' learning situation. Through big data mining and analysis, and algorithm recommendation, we can accurately grasp the characteristics of students' learning, thinking, and behavior, achieve accurate teaching, and improve the teaching effect and educational effectiveness of political thought courses.

RETRACTED

The feasible implementation strategy of AI-driven political thought teaching mode innovation is to rely on AI technology to promote political thought classes to be more quality and effective on the basis of traditional teaching. Ideological level is as follows: change ideas, face the future, and clarify the innovation goal of political thought teaching mode [35].  Figure 8 shows the research popularity of AI-driven political thought teaching mode innovation in recent years. Secondly, we will introduce the curriculum implementation standards of artificial intelligence embedded in political thought courses and formulate relevant curriculum systems and smart textbook systems. On the basis of maintaining the relative stability of the required courses of political thought courses, adjust and innovate the artificial intelligence embedded in the political thought course system, and combine the characteristics of each school to build a curriculum system of compulsory courses plus artificial intelligence political thought elective courses. Finally, improve the incentive mechanism of political thought teachers to enhance teachers' professional identity, sense of honor, and sense of responsibility. We should include outstanding members of political thought teachers in various high-level talent projects, promote the implementation of post allowance for political thought teachers according to local conditions, take political thought teachers as an important source of cadres, strengthen the publicity of advanced models, and play an exemplary and leading role. The technical level is as follows: the first step is to build an accurate political thought platform and an intelligent political thought platform. Building a smart political thought platform is a model of deeply integrating the working advantages of political thought education with advanced technology. Accurate political thought education requires accurate identification of objects and accurate prediction of their needs, targeted and accurate supply of political thought learning resources, accurate teaching, and accurate evaluation in the later stage. The second step is to build an “artificial intelligence+political thought course” reform think tank, which is composed of relevant scholars and experts in the field of political thought education and artificial intelligence. With its highly intensive intelligence attribute, this paper makes an in-depth study of the problems in the process of artificial intelligence embedded in political thought teaching from a professional perspective and puts forward relevant new ideas, new schemes, and new strategies. The third step is to lay out the research and development of key common technology system of artificial intelligence in the field of political thought education, make overall planning guidance for the research of key common technology from the national level, and increase relevant support. The following is the action level: improve the management and risk control ability of artificial intelligence, ensure the positive application of artificial intelligence in political thought teaching, and effective scientific management helps to improve the antirisk ability of artificial intelligence information technology in driving the innovation of political thought teaching mode. Improve the ability of artificial intelligence R amp D and promotion, adapt to the changes in the educational environment with technological innovation, and maintain a rational attitude towards artificial intelligence technology. It is clear that artificial intelligence information technology is not completely objective and needs to be vigilant to reduce the probability of artificial intelligence information technology risks. Improve the ability of teaching, communication, technology application, and information processing, realize the deep integration of artificial intelligence and political thought teaching, let political thought teachers receive education first, give play to teachers' enthusiasm, initiative, and creativity, make political thought teachers have high and systematic teaching ability and teaching level, and clarify their position and role.

RETRACTED

## 5. Conclusion

The overall innovation of the teaching paradigm of political thought courses in the new technology era should be based on a correct understanding of the disciplinary attributes of political thought courses. The introduction of teaching assistant robots can meet the needs of teachers' precise teaching and students' personalized learning. Using big data to continuously capture students' “classroom portraits” can achieve a sustainable analysis of the changes in the ideological status of young college students. Relying on new technology to innovate the teaching paradigm of political thought courses, we should deal with the relationship between instrumentality and humanism. Deal with the integration between the instrumentality of artificial intelligence and the value of political thought education. The core goal of political thought education is to achieve value guidance, ability improvement, and knowledge transfer. In the future, on the basis of studying and judging the specific situation of colleges and universities, we should form a situation in which political thought courses are integrated with new technologies. The deep integration of information technology and political thought education will make the above three core goals specific, so as to promote the differentiated teaching of individual students. In addition, in the process of in-depth integration, we should also constantly sum up experience, improve experience, find new problems, and solve new problems.

Political thought teachers should face up to the existence of artificial intelligence and realize that political thought courses are not unrelated to artificial intelligence. Secondly, teachers of political thought courses should grasp the fundamental purpose and requirements of political thought courses, adhere to the correct guidance, and do a good job in the basic response to artificial intelligence on this basis. A key problem here is to incorporate the frontier issues of artificial intelligence into the content of political thought courses. It is not a random extension of the teaching content aimlessly. It is not to say that you can “talk casually” or “talk nonsense” in the teaching process. In particular, you should carefully deal with some controversial new issues. Thirdly, teachers of political thought courses also need to keep pace with the times, improve their understanding of artificial intelligence, and master some knowledge and theories related to artificial intelligence in combination with the teaching purpose and content of political thought courses. Of course, political thought teachers' learning of artificial intelligence knowledge is to serve the political thought course well, so their learning does not need to master the theoretical and technical knowledge of artificial intelligence in depth but should focus on the intersection of artificial intelligence and humanities and social sciences and have a basic understanding and thinking of the frontier issues and discussions in the intersection of artificial intelligence and Humanities and social sciences. Finally, political thought teachers should actively try to integrate AI-related content into teaching and summarize and reflect on the actual effect, such as setting AI teaching topics, taking AI as the theme of practical teaching, and encouraging students to search and read articles and books related to AI.

The integration of IP courses and new technologies is not only beneficial to the teaching reform of IP courses but also beneficial to the management and construction of teachers. Under the background of new technology, the teaching reform of IP courses in colleges and universities should pay more attention to real-time and interactivity and combine the teaching mode of IP courses of artificial intelligence to help the overall improvement of teaching quality and level. Looking into the future, we should think about the integration of political thought teaching and artificial intelligence technology from the perspective of innovation, modernity, and development. The development trend of science and technology and education is intersection and integration. The great changes in the world have put forward new requirements for all political thought teachers. We should strengthen theoretical consciousness, stick to the main position of political thought teaching, and realize the unity of following the classroom rules, political thought teaching rules, and students' cognitive rules in teaching practice. We should start from the overall situation and strategic height of the development of the cause of the party and the country and cultivate new people of the times who are responsible for the rejuvenation of the nation through AI enabled political thought teaching.

RETRACTED

## Figures and Tables

**Figure 1:** About the connection between artificial intelligence, robotic learning, and deep learning.

**Figure 2:** Distribution of teaching age of political thought teachers.

**Figure 3:** Distribution of political thought teachers' cultural literacy.

**Figure 4:** Distribution proportion map of political thought teaching methods.

**Figure 5:** Subjective Bayesian method operation architecture.

**Figure 6:** The familiarity of political thought teachers with the basic principles of teaching practice.

**Figure 7:** Understanding of artificial intelligence technology to students' interests.

**Figure 8:** Research on the innovation of teaching mode of political thought courses driven by artificial intelligence.

## Data Availability

The data used to support the findings of this study are available from the corresponding author upon request.
